The article "Diagnosis of Cardiac Rehabilitation after Percutaneous Coronary Intervention in Acute Myocardial Infarction Patients by Emission Computed Tomography Image Features under Filtered Back Projection Reconstruction Algorithm" was published in 2021. Journal: J Healthc Eng.

# Diagnosis of Cardiac Rehabilitation after Percutaneous Coronary Intervention in Acute Myocardial Infarction Patients by Emission Computed Tomography Image Features under Filtered Back Projection Reconstruction Algorithm

**DOI:** 10.1155/2021/6844549

**Published:** 2021-10-22

**Authors:** Yuan Lv, Suyu Zhao

**Affiliations:** Department of Cardiology, Lishui People's Hospital, Lishui 323000, Zhejiang, China

## Abstract

This study aimed to explore the application value of emission computed tomography (ECT) imaging technology based on filtered back projection reconstruction algorithm (FBP) in cardiac function examination after percutaneous coronary intervention (PCI) in patients with acute myocardial infarction (AMI). Eighty patients with myocardial infarction diagnosed by medical history, electrocardiograph (ECG), and myocardial enzyme admitted to hospital from February 2018 to February 2019 were selected as the research objects. All patients underwent PCI seven days after the onset of myocardial infarction. ECT was performed for all patients before and after surgery. In addition, all ECT images were processed by the FBP reconstruction algorithm. On this basis, preoperative and postoperative cardiac surgery function and ischemia of the patients were diagnosed. Then, the diagnostic results were compared with the results of coronary angiography and echocardiogram. The results showed that all patients had a total of 541 segments before PCI surgery. ECT examination revealed 294 abnormal segments of the ventricular wall, with a total score of 585 points. A total of 100 segments were scored with 1 point, a total of 194 segments were scored with 2 points, and a total of 50 segments were scored with 3 points. After PCI, the number of abnormal segments was reduced to 58, with a total score of 193. There were 6 segments with a score of 1, 44 segments with a score of 2, and 5 segments with a score of 3. The left ventricular diastolic volume (EDV), left ventricular systolic volume (ESV), stroke volume (CO), and ejection fraction (EF) of the patients before the operation were 148 ± 16 mL, 77 ± 14.5 mL, 4.29 ± 0.37 L/min, and 41.9 ± 8%, respectively. The EDV, ESV, CO, and EF of the patients after surgery were 132 ± 16 mL, 62 ± 13 mL, 4.89 ± 0.71, and 53 ± 6%, respectively. Significant changes occurred in various systolic function parameters before and after surgery, *P* < 0.05. The standardized regression coefficients of the three groups were 0.32, 0.41, and 0.47, respectively, *P* < 0.05, which indicated that the greater the coronary artery stenosis rate, the higher the diagnostic coincidence rate of left anterior descending limb (LAD), left circumflex branch (LCX), and left coronary artery (RCA). The conformity of ECT imaging in the LCX group for diagnosis of myocardial ischemia was higher than that of UCG, *P* < 0.05. To sum up, the ECT technology based on the FBP reconstruction algorithm had a good application prospect in the diagnosis of cardiac function recovery in AMI patients after PCI.

The article "Diagnosis of Cardiac Rehabilitation after Percutaneous Coronary Intervention in Acute Myocardial Infarction Patients by Emission Computed Tomography Image Features under Filtered Back Projection Reconstruction Algorithm" was published in 2021. Journal: J Healthc Eng.

## 1. Introduction

In recent years, with the aggravation of the aging of the population in China and the increasing pressure on people's life, the prevalence and mortality of cardiovascular diseases are rising. Among them, coronary atherosclerotic heart disease (CAD) has become one of the primary cardiovascular diseases threatening the life and health of Chinese people [1]. Coronary heart disease (CHD) is defined as a narrowing or obstruction of the lumen caused by atherosclerosis of the coronary artery, or a functional change in the coronary artery that leads to myocardial ischemia, hypoxia, or necrosis that further leads to heart disease. Clinically, CHD is generally classified into five types: (i) asymptomatic myocardial ischemia, (ii) angina pectoris, (iii) acute myocardial infarction (AMI), (iv) ischemic cardiomyopathy, and (v) sudden death. Among them, AMI is the most common and serious [2]. AMI is defined as the rapid reduction or interruption of the blood supply of the coronary artery based on coronary artery disease, resulting in severe and persistent acute ischemia of the corresponding myocardium leading to myocardial necrosis. Once myocardial infarction occurs, ventricular remodeling will occur, which will further lead to complications such as left ventricular dysfunction and congestive heart failure. They will seriously affect the long-term prognosis of patients and reduce the quality of life of patients [3]. Effective and timely reperfusion is the key to the early treatment of AMI. Clinical data showed that percutaneous coronary intervention (PCI) has a good therapeutic effect on AMI. However, recent studies pointed out that PCI has time compliance in the treatment of AMI. Direct PCI within twelve hours of acute myocardial infarction can effectively save the myocardium, reduce the size of myocardial infarction, and improve left ventricular remodeling. However, PCI was less effective in saving dying cardiomyocytes after seven days of acute myocardial infarction. Its effects on improving the blood flow of the left ventricular remodeling, resting or hibernating myocardium, and preventing the expansion and extension of the infarct area remain controversial. In addition, many studies revealed that about 30%∼40% of AMI patients will have no-reflow after PCI, which seriously affects the therapeutic effect and leads to the prognosis of patients. Therefore, there is an urgent need for an effective method to examine and evaluate the cardiac function recovery of AMI patients after PCI [4–6].

The article "Diagnosis of Cardiac Rehabilitation after Percutaneous Coronary Intervention in Acute Myocardial Infarction Patients by Emission Computed Tomography Image Features under Filtered Back Projection Reconstruction Algorithm" was published in 2021. Journal: J Healthc Eng.

Radionuclide emission computed tomography (ECT) is a computer aided technique, which uses isotopes to label drugs, thereby measuring the concentration intensity of isotopes in various organs in the body and its change with time based on the principle of human body synthesis. In this way, the visual shape of the organs is displayed, and the functional image information of their physiological process and metabolism is reflected [7]. ECT technology develops rapidly and has become one of the markers of nuclear medicine modernization at present [8]. It has been widely used in the diagnosis of tumors, bone diseases, and cerebrovascular diseases because it can well combine functional images with anatomical images. It is also the main means of heart disease diagnosis, especially in the diagnosis of coronary heart disease, which shows a good diagnostic efficiency and has become one of the recognized methods to detect coronary heart disease. When radiopharmaceuticals enter the coronary arteries, they are selectively ingested by normal cardiomyocytes, and the amount ingested is proportional to the coronary blood flow. When a coronary artery is narrowed or blocked, blood flow in the coronary arteries is reduced, and heart muscle cells are damaged. At that point, the ability of the heart muscle to absorb radioactive drugs is reduced or even unable to absorb them. Therefore, ECT can accurately display the metabolism and blood flow of the myocardium, so as to further determine whether the myocardium is ischemic, ischemic site, and ischemic area. Compared with coronary angiography, exercise plate, and other examination methods, it has the advantages of noninvasive and no exercise load, so it is a relatively safe and effective examination method in clinical practice [9]. Patients with negative ECT examinations can basically exclude coronary heart disease. For patients with positive ECT examination, the specific coronary artery lesions are further inferred according to the abnormal blood flow distribution and perfusion volume.

ECT examination is mainly classified into functional image examination and anatomical structure image examination, but the image resolution collected by functional image examination is very low and lacks anatomical information. To solve this problem, image fusion is proposed. At present, CET and CT can be organically combined to provide high-quality images with anatomical localization. To a certain extent, the quality of ECT images is provided [10]. However, there are still many problems such as image quality distortion caused by attenuation factors such as the Compton effect and scattering on image fusion. Image reconstruction technology has developed rapidly in recent years. According to the collected data, the image is reconstructed by computing the pixels in the image matrix. FBP is the most widely used algorithm in image reconstruction at present. At present, it mainly exists in the X-ray CT system, but there are few studies on its application in CET [11].

The article "Diagnosis of Cardiac Rehabilitation after Percutaneous Coronary Intervention in Acute Myocardial Infarction Patients by Emission Computed Tomography Image Features under Filtered Back Projection Reconstruction Algorithm" was published in 2021. Journal: J Healthc Eng.

In this study, patients with acute heart infarction were taken as the research objects. ECT examination was performed before and after PCI. FBP algorithm was used to process the obtained images, and on this basis, the efficacy of PCI in MAI was evaluated, to provide reference and basis for clinical use of ECT, PCI, and FBP algorithm in treatment and diagnosis of AMI.

## 2. Materials and Methods

### 2.1. Research Objects

A total of 80 patients admitted to the hospital from February 2018 to February 2019 who were diagnosed with AMI by medical history, ECG, and myocardial enzyme were selected. There were 55 male patients and 25 female patients, with an average age of 61.6 ± 11.2 years. Exclusion criteria are as follows: patients with onset less than twelve hours or longer than one month; patients suffering from cerebrovascular diseases or severe liver and kidney dysfunction or hyperthyroidism; patients suffering from malignant arrhythmia, congenital heart disease, cardiac hypertrophy, and myocarditis resulting in cardiac insufficiency; patients with a history of respiratory dysfunction, malignant tumor, or active bleeding; and patients who were long-term bedridden and unable to perform ECT examination. All studies had obtained patients' informed consent and met the requirements of medical ethics.

### 2.2. Overview of Research Methods

All the subjects underwent percutaneous coronary intervention (PCI) seven days after myocardial infarction. All patients were examined with radionuclide emission computed tomography (ECT) before and after surgery. All ECT images are processed by filtering back projection reconstruction algorithm. On this basis, the preoperative and postoperative cardiac operation function and ischemia were diagnosed. The diagnostic results were compared with coronary angiography and ultrasound ECG.

### 2.3. ECT Inspection Method

The inspection instrument was Siemens symbia-1, the imaging agent was 9mTc-MIBI, and the radiochemical purity was >95%. All patients were routinely given antiplatelet aggregation, anticoagulants, beta-blockers, nitrates, ACEI drugs, and statins after admission. 99mTc-MIBI was intravenously injected on the morning of the 7th day of admission, in the fasting and resting state, with a dose of 925∼1110 MBq (25∼30 mCi). Half an hour later, the patient was fed a fried egg or 250 mL of pure milk. Resting-gated myocardial perfusion imaging was performed 1.5 to 2 hours later. ECT was equipped with a parallel hole low energy and high-resolution collimator. The R wave of ECG was the trigger wave. The patient lied on the examination bed with his head outwards. ECG gating device was opened, and the ECG electrodes were connected correctly. The starting angle of probe 1 was −45°, and the starting angle of probe 2 was 56°. The angle between probes was 101°, one position per 3D, running 1050 in total, and 36 individual positions were collected. Eight frames were collected per cardiac cycle, and the acceptable heart rate range was ±20% of the mean heart rate. The matrix was 64 × 64, and the acquisition time was 30 seconds/section. The energy peak was 140, and the magnification (ZOOM) was 1.33.

The article "Diagnosis of Cardiac Rehabilitation after Percutaneous Coronary Intervention in Acute Myocardial Infarction Patients by Emission Computed Tomography Image Features under Filtered Back Projection Reconstruction Algorithm" was published in 2021. Journal: J Healthc Eng.

ECT results were classified into four grades: normal (grade 0), decreased perfusion (grade 1), substantially decreased perfusion (grade 2), and perfusion defect (grade 3). The calculation of wall thickening rate was automatically graded into normal wall thickening rate (>25%, grade 0), reduced (10∼24%, grade 1), substantially reduced (10% to 9%, grade 2), and substantially reduced or no exercise (<9%, grade 3).

### 2.4. Image Processing Method

The back projection reconstruction algorithm usually introduces star artifacts, which will lead to image distortion after reconstruction. This problem can be solved by rate-wave processing of the image before reconstruction.

The projection theorem is the basis of image reconstruction. The specific content is as follows. A slice of the 2D Fourier transform $F\left(w_{1},w_{2}\right)=\hat{F}\left(\rho ,\phi \right)$ of *f*(*x*, *y*) is given by the 1D Fourier transform of an image *p*_*ϕ*_(*x*_*r*_) projected at the angle *ϕ* of view *f*(*x*, *y*). The slice and the axis *w*_1_ intersect at an angle *ϕ* and pass through the origin of the coordinate. The specific schematic diagram is shown in Figure 1. It is further explained that the 1D Fourier transform of the projection of the image *f*(*x*, *y*) in the direction *ϕ* gives a slice of the 2D Fourier transform of *f*(*x*, *y*), and the position of the slice passes through the origin and forms an angle *ϕ* with *w*_1_.

(1) $$\begin{array}{c} \zeta_{1}\left[p_{\phi }\left(x_{r}\right)\right]={\hat{F}\left(\rho ,\phi \right)|}_{\phi =arctgw_{2}/w_{1}}. \end{array}$$

The relationship between the projection angle *ϕ* of view and the rotation coordinates (*x*_*r*_, *y*_*r*_) and (*x*, *y*) is as follows.

(2) $$\begin{array}{c} \left\{\begin{array}{c} x_{r}=x\;\cos\;\phi +y\;\sin\;\phi ,\\ y_{r}=-x\;\sin\;\phi +y\;\cos\;\phi . \end{array}\right. \end{array}$$

*w*_1_, *w*_2_ are not independent but bound by

(3) $$\begin{array}{c} \left\{\begin{array}{c} w_{1}=2\pi \rho \;\cos\;\phi ,\\ w_{2}=2\pi \rho \;\sin\;\phi . \end{array}\right. \end{array}$$

FBP reconstruction is as follows. The image to be built is *a*(*x*, *y*); then, its 2D Fourier transform is $A\left(w_{1},w_{2}\right)=\hat{A}\left(\rho ,\theta \right)$. According to the central slice theorem, $\hat{A}\left(\rho ,\theta \right)$ is obtained by 1D Fourier transform of *p*_*ϕ*_(*x*_*r*_) of the projection of *a*(*x*, *y*) under different viewing angles, which is expressed as follows.

(4) $$\begin{array}{c} A\left(w_{1},w_{2}\right)=\hat{A}\left(\rho ,\theta \right)=\xi_{1}\left[p_{\phi }\left(x_{r}\right)\right]=P_{\phi }\left(\rho \right)=P\left(\rho ,\phi \right). \end{array}$$

The image to be built is as follows.

(5) $$\begin{array}{c} \overset{\Delta }{a}\left(r,\theta \right)=a\left(x,y\right)=\xi_{2}^{-1}\left[A\left(w_{1},w_{2}\right)\right]. \end{array}$$

Then, there is

(6) $$\begin{array}{c} \overset{\Delta }{a}\left(r,\theta \right)=\int_{0}^{X}\text{d}\phi \int_{-\infty }^{\infty }\left|\rho \right|P\left(\rho ,\phi \right)e^{J\pi \rho r\;\cos\left(\theta -\phi \right)}\text{d}\rho . \end{array}$$

The second integral of equation (6) is as follows.

(7) $$\begin{array}{c} \int_{-\infty }^{\infty }\left|\rho \right|P\left(\rho ,\phi \right)e^{J2\pi \rho rcos\left(\theta -\phi \right)}d\rho . \end{array}$$

The above equation is rewritten as the inverse Fourier variant with the spatial variable *x*_*r*_ as follows.

(8) $$\begin{array}{c} \int_{-\infty }^{\infty }\left|\rho \right|P\left(\rho ,\phi \right)e^{J2\pi \rho r\;\cos\left(\theta -\phi \right)}d\rho =\int_{-\infty }^{\infty }\left|\rho \right|{P\left(\rho ,\phi \right)e^{J2\pi \rho r\;\cos\left(\theta -\phi \right)}|}_{xr=r\;\cos\left(\theta -\phi \right)},\\ =g\left[r\;\cos\left(\theta -\phi \right),\phi \right] \end{array}$$

(9) $$\begin{array}{c} g\left(x_{r},\phi \right)=p\left(x,\phi \right)*h\left(x_{r}\right). \end{array}$$

Equation (9) is substituted in equation (5), and then, equation (10) is obtained.

(10) $$\begin{array}{c} \overset{\Delta }{a}\left(r,\theta \right)=\int_{0}^{X}g\left[r\;\cos\left(\theta -\phi \right),\phi \right]\text{d}\phi . \end{array}$$

Equation (10) is the filter back projection equation, which can reflect the various steps of the filter back projection algorithm. The schematic block diagram of the specific filtering back projection reconstruction process is shown in Figure 2. Generally speaking, it has three major steps:

- The projection *p*(*x*_*r*_, *ϕ*_*i*_) measured under the fixed viewing angle *ϕ*_1_ is filtered to obtain the filtered projection *g*(*x*_*r*_, *ϕ*_*i*_)
- For each *ϕ*_*i*_, *g*(*x*_*r*_, *ϕ*_*i*_) is projected back on all points (*r*, *θ*) on the ray satisfying *x*_*r*_=*r*  cos(*θ* − *ϕ*_*i*_)
- All the back projection values (0 < *ϕ* < *π*) in the second step are integrated to get the reconstructed image

The article "Diagnosis of Cardiac Rehabilitation after Percutaneous Coronary Intervention in Acute Myocardial Infarction Patients by Emission Computed Tomography Image Features under Filtered Back Projection Reconstruction Algorithm" was published in 2021. Journal: J Healthc Eng.

### 2.5. Image Reconstruction Effect Evaluation

The required calculation is used to evaluate the reconstruction effect of the algorithm proposed in this study and the traditional algorithm. The lower the amount of calculation, the better the reconstruction effect. The specific calculation process is as follows. It is supposed that the one-dimensional calculation of *N* points in the algorithm proposed in this study is a function of the transformation length IV, denoted by *A*(*N*), and *A*(*N*)=*O*(*N*  log_2_  *N*). The calculation amount of the first step of filtering is real number multiplication and addition of *A*(2*N*) times. The calculation amount of the second step is real number multiplication of 2*N* times. The calculation amount of the third step is the same as that of the first step. Therefore, to complete the filtering of azimuth projection data, the amount of calculation required is expressed as follows.

(11) $$\begin{array}{c} \left\{\begin{array}{c} \text{Real number multiplication: }2A\left(2N\right)+2N,\\ \text{Real number addition: }2A\left(2N\right). \end{array}\right. \end{array}$$

The calculation steps required by the traditional algorithm are the same as those of the new method as follows.

(12) $$\begin{array}{c} \left\{\begin{array}{c} \text{Real number multiplication: }5A\left(2N\right)+4N,\\ \text{Real number addition: }5A\left(2N\right). \end{array}\right. \end{array}$$

### 2.6. Treatment Methods

All patients underwent PCI seven days after AMI. 6F guiding catheter was placed at the opening of the diseased vessel. The guidewire was inserted to the distal end of the stenosis and the occlusion. Balloon angioplasty was performed on the lesion site through balloon insertion along the guidewire. Then, according to the diameter and length of the lesion, the appropriate stent was selected for intracoronary stent implantation, and the balloon pressure of the stent was preexpanded and the balloon pressure of the stent was released regarding the characteristics of the lesion. All patients received 9mTc-MIBI resting-gated myocardial perfusion two days after PCI, using the same method as before. The myocardial perfusion and cardiac function improvement were evaluated. The imaging method was the same as before. To ensure the comparability of myocardial images, the activity of the imaging agent, the instrument, and the position of the patient were as consistent as possible before and after stent implantation in the same patient.

The article "Diagnosis of Cardiac Rehabilitation after Percutaneous Coronary Intervention in Acute Myocardial Infarction Patients by Emission Computed Tomography Image Features under Filtered Back Projection Reconstruction Algorithm" was published in 2021. Journal: J Healthc Eng.

### 2.7. Statistical Methods

SPSS 11.0 was employed for data statistics and analysis. Mean ± standard deviation (□*x* ± *s*) was how measurement data were expressed, and the *t*-test was used to test the significance of patients' data before and after the operation. Percentage (%) was how count data were expressed, and the *χ*^2^ test was used to test the significance. The pairwise comparison was performed by analysis of variance. The difference was statistically considerable with *P* < 0.05.

## 3. Results

### 3.1. General Patient Information

General information of the patient's age and sex, smoking history, number of diseased blood vessels, coronary artery branches, and ECG are shown in Tables 1 and 2. The average age of the patients was 59.1 ± 12.33. There were 55 male patients, accounting for 68.7%. The number of patients with diseased blood vessels of 1 and 2 was 37 and 38, respectively. The numbers of patients with the three types of coronary artery branch lesions were basically the same, which were 36, 27, and 31, respectively. Most of the patients showed AMI and myocardial ischemia.

### 3.2. Patient ECT Examination Results

The ECT examination results before and after the operation and the comparison of ECT before and after processing by the FBP reconstruction algorithm are shown in Figures 3 and 4. The results of ECT examination before PCI operation indicated that the left ventricular apex, anterior wall, and septal segment were almost defective in resting state, and the inferior wall partial septal segment was obviously sparse or defective. Cardiac perfusion and filling gradually recovered over time after PCI surgery. Figures 3 and 4 were compared, the quality of the ECT image processed by the unfiltered back projection reconstruction algorithm was poor, and the image was blurry. After being processed by the FBP reconstruction algorithm, the image quality was substantially improved, and the contour and edge of the target observation part became clearer.

### 3.3. Comparison of the Amount of Calculation Required for Image Reconstruction of the Two Algorithms

Table 3 shows the comparison results of the calculation amount required for image reconstruction under different algorithms. In the new method, since only [*M*/4] back projection calculations of azimuths require positioning operations [*X*] (representing the smallest integer greater than *X*), and in each direction, only the pixels in the positioning part need positioning operations, the calculation amount of multiplication in the new method operation is 3*N*[*M*/4]/2 approximately, and the calculation amount of other operations can be deduced by analogy. Therefore, the required calculation of the new method is only 1/8 of the traditional method.

The article "Diagnosis of Cardiac Rehabilitation after Percutaneous Coronary Intervention in Acute Myocardial Infarction Patients by Emission Computed Tomography Image Features under Filtered Back Projection Reconstruction Algorithm" was published in 2021. Journal: J Healthc Eng.

### 3.4. Comparison of Myocardial Perfusion before and after PCI

The comparison of myocardial perfusion in patients before and after PCI operation is shown in Figure 5. All patients had a total of 541 segments before PCI. ECT examination revealed 294 abnormal segments of the ventricular wall, with a total score of 585 points. A total of 100 segments were scored with 1 point, a total of 194 segments were scored with 2 points, and a total of 50 segments were scored with 3 points. After PCI, the number of abnormal segments was reduced to 58, with a total score of 193. There were 6 segments with a score of 1, 44 segments with a score of 2, and 5 segments with a score of 3. The decrease in blood perfusion of patients after PCI surgery was considerable.

### 3.5. Comparison of Systolic Function Parameters of Patients before and after PCI

The comparison of the cardiac function parameters of the patients before and after PCI is shown in Figure 6. The EDV, ESV, CO, and EF of the patients before the operation were 148 ± 16 mL, 77 ± 14.5 mL, 4.29 ± 0.37 L/min, and 41.9 ± 8%, respectively. The EDV, ESV, CO, and EF of the patients after surgery were 132 ± 16 mL, 62 ± 13 mL, 4.89 ± 0.71, and 53 ± 6%, respectively. Various parameters of cardiac systolic function changed substantially before and after the operation, and the difference was considerable, *P* < 0.05.

### 3.6. Comparison of ECT Imaging and CAG Results Based on FBP Reconstruction Algorithm

According to the classification of coronary artery disease, the patients were rolled into three groups of left anterior descending limb (LAD), left circumflex artery (LCX), and left coronary artery (RCA), to perform regression analysis of ECT diagnosis coincidence rate and coronary artery stenosis rate. From Figure 7, in the LAD group, *F* = 4.39, *P* < 0.05, which was statistically considerable. In the LCX group, *F* = 8.21, *P* < 0.05, which was statistically considerable. In the RCA group, *F* = 11.36, *P* < 0.05, which was statistically considerable. The standardized regression coefficients of the three groups were 0.29, 0.42, and 0.48, respectively, and the significance of the three groups was *P* < 0.05, which indicated that the greater the coronary artery stenosis rate, the higher the diagnostic coincidence rate of the three groups of LAD, LAD, and RCA.

### 3.7. Comparison of Diagnosis Coincidence between Myocardial ECT Imaging and UCG

The comparison results of myocardial ECT imaging and UCG diagnosis are shown in Figure 8. There was no difference between the LAD group's myocardial ECT imaging in the diagnosis of myocardial ischemia and UCG, *P*=1. The conformity of ECT imaging in the LCX group for diagnosis of myocardial ischemia was higher than that of UCG, and the difference was considerable, *P* < 0.05. The conformity of ECT imaging in the RCA group for diagnosis of myocardial ischemia was higher than that of UCG, but the difference was not considerable, *P* > 0.05.

The article "Diagnosis of Cardiac Rehabilitation after Percutaneous Coronary Intervention in Acute Myocardial Infarction Patients by Emission Computed Tomography Image Features under Filtered Back Projection Reconstruction Algorithm" was published in 2021. Journal: J Healthc Eng.

## 4. Discussion

AMI refers to the rapid reduction and interruption of the blood supply of the coronary artery when the coronary artery disease occurs, and then, the relevant myocardium presents continuous ischemia and then leads to myocardial necrosis [12]. As the most serious coronary heart disease, acute attack infarction seriously threatens people's life and health. In addition, the aging of our population is becoming more and more serious. AMI has become one of the major causes of death in China. Currently, the most effective treatment for AMI is PCI [13]. All the patients in this study underwent PCI seven days after the occurrence of AMI, and the cardiac perfusion function of most patients was improved after the operation. Then, the parameters of cardiac systolic function all changed greatly compared with those before the operation, which suggested that PCI had a good effect on cardiac perfusion and systolic function in patients with AMI.

At present, coronary angiography is still the gold standard for the diagnosis of AMI. With the continuous development of nuclear medicine and imaging technology, radionuclide ECT has also been applied in the diagnosis of heart diseases [14]. ECT is defined as a computer aided technology that uses isotopes to label drugs. Using the principle of human body synthesis, it measures the concentration intensity of isotopes in various organs of the body and its change with time. In this way, the visual shape of the organs is displayed and the functional image information of their physiological process and metabolism is reflected [15]. Clinical data showed that ECT can well reflect myocardial metabolism and blood flow. ECT can also judge the bleeding site, whether bleeding or not, and bleeding area. Compared with coronary angiography, exercise plate, and other examination methods, it has the advantages of noninvasive and no exercise load, which is a noninvasive examination method with good clinical application prospects at present. However, there is currently no consensus on the accuracy, sensitivity, and specificity of ECT in the diagnosis of AMI [16].

The article "Diagnosis of Cardiac Rehabilitation after Percutaneous Coronary Intervention in Acute Myocardial Infarction Patients by Emission Computed Tomography Image Features under Filtered Back Projection Reconstruction Algorithm" was published in 2021. Journal: J Healthc Eng.

Image reconstruction is an important research branch in image processing. It refers to the reconstruction of images based on the data obtained from object detection. Its significance lies in obtaining the image of the internal structure of the detected object without causing any physical damage to the object. Due to its considerable advantages, it has shown unique importance in various application fields [17–19]. For example, it has many applications in medical radiology, nuclear medicine, electron microscopy, radio radar astronomy, light microscopy, holographic imaging, and theoretical vision. FBP algorithm is one of the most widely used algorithms in medical image reconstruction. At present, it is widely used in the generation X-ray CT system [20–22]. CT examination is an important part of the ECT examination. In addition, the images obtained by CT examination are generally of poor quality and low resolution, which seriously affects the quality of the final ECT image fusion. In addition, the images obtained by ECT examination are all the images obtained by the fusion of CT examination and radiological examination, which is also one of the reasons that affect the image quality of ECT examination. At present, the application research of the FBP reconstruction algorithm is basically focused on CT and X-ray image processing, while the application research of ECT image processing is almost absent [23–26].

In this study, the diagnostic effect of ECT image features based on the FBP reconstruction algorithm on the recovery of cardiac function in patients with AMI after PCI surgery was explored. The results showed that all patients had a total of 541 segments before PCI. ECT examination showed 294 abnormal segments of the ventricular wall, with a total score of 585. A total of 100 segments were scored as 1 point, a total of 194 segments were scored as 2 points, and a total of 50 segments were scored as 3 points. After PCI, the abnormal segments were reduced to 58 segments, with a total score of 193. Six segments scored 1 point, 44 segments scored 2 points, and 5 segments scored 3 points. The preoperative EDV, ESV, CO, and EF were 148 ± 16 mL, 77 ± 14.5 mL, 4.29 ± 0.37 L/min, and 41.9 ± 8%, respectively. The EDV, ESV, CO, and EF of the postoperative patients were 132 ± 16 mL, 62 ± 13 mL, 4.89 ± 0.71, and 53 ± 6%, respectively. All systolic function parameters changed significantly after the operation, *P* < 0.05. The standardized regression coefficients of the three groups were 0.32, 0.41, and 0.47, respectively, *P*=0.05, indicating that the greater the coronary stenosis rate, the higher the diagnostic coincidence rate of LAD, LAD, and RCA. The diagnostic conformity of ECT images in the LCX group for myocardial ischemia was higher than that of UCG, *P* < 0.05, which showed that the results of ECT examination after PCI showed that the patient's cardiac perfusion and cardiac systolic function were greatly improved. The coincidence rate of the ECT examination based on the filtered back projection reconstruction algorithm for the cardiac function examination results and the coronary angiography examination results increased with the increase of the coronary artery stenosis rate. Compared with cardiac ultrasound, the ECT examination based on the filtered back projection reconstruction algorithm had a higher degree of agreement between the results of the cardiac function examination and the results of coronary angiography. In summary, the ECT technology based on the filtered back projection reconstruction algorithm had a good application prospect in the examination of cardiac function after PCI in AMI patients. However, due to the limited sample size and space, the study was not comprehensive and in-depth enough. In future studies and work, the sample will be further expanded and further studied.

The article "Diagnosis of Cardiac Rehabilitation after Percutaneous Coronary Intervention in Acute Myocardial Infarction Patients by Emission Computed Tomography Image Features under Filtered Back Projection Reconstruction Algorithm" was published in 2021. Journal: J Healthc Eng.

## 5. Conclusion

This study investigated the diagnostic effect of ECT image features based on the FBP reconstruction algorithm on cardiac recovery after PCI in AMI patients. The results showed that the patients' visceral function recovered significantly after PCI, and ECT based on the FBP reconstruction algorithm had better performance in cardiac function examination than cardiac ultrasound. This study provides a reference and basis for the application of PCI, FBP reconstruction algorithm, and ECT in the diagnosis and treatment of AMI patients. However, due to the limited sample size and space, this study still has some limitations and deficiencies. In future studies and work, we will expand the sample size to further study this problem.

## Figures and Tables

**Figure 1:** Coordinate system used for FBP.

**Figure 2:** Schematic diagram of FBP reconstruction.

**Figure 3:** ECT images of patients at various stages before processing by the FBP reconstruction algorithm.

**Figure 4:** ECT images of patients at various stages after processing by the FBP reconstruction algorithm.

**Figure 5:** Classification of ECT examination results before and after surgery.

**Figure 6:** Comparison of patient's systolic function before and after surgery, compared with before operation, ^*∗*^*P* < 0.05.

**Figure 7:** Regression analysis of ECT diagnosis coincidence rate and coronary artery stenosis rate.

**Figure 8:** Comparison of the diagnosis coincidence between myocardial ECT imaging and UCG.

**Table 1:** Patient age and underlying disease data.

Index	*N* = 80
Age (years)	59.1 ± 12.33
Gender (male, *n* (%))	55 (68.7%)
Smoking history (*n* (%))	53 (66%)
Hypertension (*n* (%))	44 (55%)
Diabetes mellitus (*n* (%))	77 (96.2%)
Dyslipidemia (*n* (%))	61 (76.25%)

The article "Diagnosis of Cardiac Rehabilitation after Percutaneous Coronary Intervention in Acute Myocardial Infarction Patients by Emission Computed Tomography Image Features under Filtered Back Projection Reconstruction Algorithm" was published in 2021. Journal: J Healthc Eng.

**Table 2:** UCG examination and coronary artery lesions of patients.

Item		Case number
Number of diseased vessels	0	9
	1	37
	2	38
	3	11
Types of coronary artery branch lesions	LAD	37 (46%)
	LCX	26 (32.5%)
	RCA	31 (38.7%)
Echocardiographic test results	Normal	2 (2.5%)
	Myocardial ischemia	39 (48.75%)
	Myocardial infarction	39 (48.75%)

**Table 3:** The amount of calculation required for reconstruction under different algorithms.

Operation	Multiplication	Addition	Rounding
Algorithm			
Traditional algorithm	3*MN*	2*MN*^2^	*MN* ^2^
New method	3*N*[*M*/4]/2	*N* ^2^[*M*/4]	*N* ^2^[*M*/4]/2

## Data Availability

The data used to support the findings of this study are available from the corresponding author upon request.
